# Study on the Influencing Factors and Willingness to Pay of Consumers Purchasing Ecological Agricultural Products

**DOI:** 10.1155/2022/8469996

**Published:** 2022-09-12

**Authors:** Huicheng Hao, Sixuan Yin, Hang Yu, Zemin Liu, Ziyu Liu

**Affiliations:** ^1^College of Engineering, Northeast Agricultural University, Heilongjiang Province, China; ^2^Beijing, School of Economic and Management, Beijing Forestry University, China

## Abstract

With the steady rise of China's agricultural production and management level, the market of ecological agricultural products has developed rapidly, and consumers are increasingly concerned about ecological agricultural products. Consumers' cognition and purchase intention are the keys to determine their future development. This research is aimed at ensuring that consumers have access to high-quality ecological agricultural products, thereby promoting the supply and production of ecological agricultural products, minimizing agricultural carbon emissions, and providing information on sustainable food pricing. Based on the research status at home and abroad, this study combines the questionnaire survey method to study the influencing factors and willingness to pay of consumers purchasing ecological agricultural products. A total of 601 online questionnaires from consumers in Harbin, a city in northeastern China, were collected, and statistical factor analysis, principal component analysis, and regression analysis were used to study the influencing factors of consumers' purchase of ecological agricultural products from both positive and negative aspects, and in-depth analysis of the reasons why consumers refuse to pay, get the most real willingness to pay and related influencing factors, and quantify the influence of various variables on consumers' purchasing behavior was done. On this basis, a logit model of survival analysis is constructed to study the premium payment level of consumers for ecological agricultural products, and the payment premium is 24.95%. The research results show that married, who have purchased ecological agricultural products, the higher the understanding of ecological agricultural products, the consumers who buy ecological agricultural products in farmers' markets, Meituan and community group purchases, and the households with higher monthly consumption of agricultural products have a significant positive correlation with consumers' purchase of ecological agricultural products. The higher the education level, the older the age, and the larger the family size were significantly negatively correlated with consumers' purchase of ecological agricultural products.

## 1. Introduction

As a large agricultural country, China is a world leader in the quantity and variety of agricultural products [1], and the scale of production and trade is expanding [2], but in terms of modern market demand, consumers are paying more attention to quality, appearance, branding, and additional services [3, 4] and are particularly concerned about the nutritional health of agricultural products [5]. In recent years, against the background of the Chinese government's support for agriculture, farmers and rural areas in order to support the development of agriculture, improve the economic income and living standards of farmers, and promote the sustainable development of rural areas [6], the rapid development and rapid rise of ecological agricultural products possesses a strong foundation for agricultural development and a greater potential for development. Ecological agricultural products refer to agricultural development mode of intensive management under the premise of protecting and improving the agricultural ecological environment, following the laws of ecology and ecological economics, using system engineering methods and modern science and technology, and producing agricultural products that meet the quality and safety requirements of agricultural products, harmless, nutritious, and healthy. In 2021, China's organic food certification area has reached 5464887.32 hectares. At present, the market of ecological agricultural products is gradually expanding, and there are more and more kinds of ecological agricultural products, and consumers have a greater demand for ecological agricultural products because they are good for health. However, the production of ecological agricultural products is relatively low compared with general agricultural products, and the sales price is higher than that of ordinary agricultural products. For this reason, it is necessary to understand the market demand of ecological agricultural products, which is conducive to the continuous improvement of the value of ecological agricultural products, bringing greater income and also contributing to energy saving and emission reduction.

Currently, agricultural products research is focused on low-carbon agricultural products [7, 8], organic agricultural products, food safety [9], quality edible agricultural products [10], and the impact of sustainable agricultural products on environmental change [11, 12]. Vinholis et al. [13] based on a survey sample of 175 farmers in the state of São Paulo, Brazil, through the Joint Cube System (SES) to assess the impact of the mesocosm system on farmers' decision to adopt an integrated crop-livestock system (ICLS) and farm performance. Increasing population and economic growth have led to an increased carbon footprint, and the level of carbon emissions varies significantly across regions [14]. Chen et al. [15] embedded ecological benefits in the policy objectives of economic efficiency-oriented agricultural production and introduced the carbon and nitrogen cycle into the life cycle evaluation theory, which led to a significant reduction in the uncertainty of carbon footprint accounting methods. Lam et al. [16] analyzed the main issues affecting agricultural land conversion, freshwater scarcity, and soil quality in the Chinese agricultural production process and studied some of the increased demand to meet the consumption of animal products in the Chinese diet. Experimental results by Gomez et al. [17] showed the great potential of new nanoagrochemicals to significantly increase crop yields while reducing the environmental impact of traditional agrochemicals, and Loo et al. [18] investigated consumers' willingness to purchase organic chicken meat in terms of healthiness, price, and purchasing channels. Żakowska-Biemans [19] conducts research on the food-related lifestyles of Polish consumers and their relationship to organic food consumption, analyzing the barriers for consumers to purchase organic food. Sánchez-Bravo et al. argue that young consumers are often perceived as being at the forefront of sustainability issues [20]. Laureati studies the determinants of children's preference and consumption of healthy foods [21]. The reasons for purchasing organic produce are diverse, and consumers who do not have a good understanding of the true characteristics of organic produce are influenced by its labeling and thus their willingness to purchase [22]. Veelen [23] investigates the impact of the financial sector and the environment on agricultural production by combining the concept of “green finance” with low-carbon agricultural products. The impact of the environment on agricultural production. Policymakers who want to increase organic consumption as an element of sustainable development need to address the key issue of price, which is a major barrier to expanding demand from current and future organic consumers [24]. However, the pricing of organic food is a multifaceted and even paradoxical issue [25], where consumers desire low prices while possibly defining them as a hint of suboptimal quality. Price plays an important role in consumer purchasing behavior, depending on the economic context, price awareness and sensitivity, trade-offs between price and value, and willingness to pay (WTP) [26]. However, while studies related to organic and low-carbon agricultural products exist in the market, there is little research on ecological agricultural products in China and a lack of comprehensive scientific studies and in-depth analysis of their current status; therefore, consumer needs are not yet fully understood. In order to stimulate the sale of ecological agricultural products, it is necessary to understand consumers' needs, influencing factors, and willingness to pay in order to provide a basis for decision making on price and sales strategies.

By studying the influencing factors and willingness to pay of consumers' purchase of ecological agricultural products, this paper believes that the core of consumers' purchase is health value and environmental value. With the frequent occurrence of food safety accidents in China, the basic requirement that consumers are willing to pay a premium for is the health and safety brought by its high quality [27, 28]. Seubelt et al. also found that price is a major factor in food choice from a sustainability perspective [29]. At the same time, environmental value is also the main reason why consumers consider purchasing ecological agricultural products. Buying ecological agricultural products can effectively promote the sustainable and healthy development of ecological agricultural products and help reduce agricultural carbon emissions.

Based on the research of other scholars and the actual situation of Chinese consumers, this study divides the factors influencing consumers' purchasing behavior of ecological agricultural products into five parts: demographic characteristics, awareness of ecological agricultural products and purchasing channels, factors influencing the purchase of ecological agricultural products, and consumers' purchasing experience and willingness to pay. Through statistical analysis of data in these five areas, key factors influencing consumers' purchase of ecological agricultural products were identified. We collected basic research data through questionnaires, applied statistical theory to test the reliability and validity of the collected data, conducted factor analysis and regression analysis on the influencing factors and came up with the degree of influence of each variable factor on consumers' purchasing behavior, and quantified the consumers' willingness to pay premium for purchasing ecological agricultural products through CVM method. The study of these factors will have important practical significance for the sustainable development of ecological agricultural products and can provide decision support for the market pricing of ecological agricultural products.

## 2. Theoretical Background

Consumers' willingness to pay is the personal evaluation of consumers for a specific commodity with a strong subjective evaluation. Consumers are the final purchasers and monetary payers of agricultural products, if ecological agricultural products want to achieve the desired market effect should be based on the establishment of consumer-centered modern marketing concept, many foreign scholars have studied the demand system of agricultural products from the perspective of consumers' willingness to pay. Market research has been conducted to understand consumer demand and purchasing power of agricultural products to explore consumer demand and willingness to pay for organic agricultural products [28, 30, 31]. Among others, it was assessed that education level may also influence consumers' awareness of environmental issues and attitudes towards the processing of ecological information [32]. Verbeke and Ward [33] studied consumers' attitudes towards EU food labeling and found information that consumers are more sensitive to labeling information. Pieniak et al. [34], through a study in the autonomous community of Aragon, Spain, separately investigated the attitudes of consumers and retailers towards beef traceability system and labeling, and the results illustrated that different participants had significantly different attitudes towards beef traceability system. The level of consumers' willingness to pay for low-carbon attributes of food products was explored using the example of low-carbon rice selected in a central Chinese city [6]. Zhang et al. proposed practical solutions to reduce the cost of agricultural products by analyzing the factors that significantly affect the willingness to purchase and payment levels of low-carbon vegetables [35].

Some typological or consumer segmentation studies [36, 37] and consumer behavior models are also common [33, 38–42]. Ma et al. conducted an empirical study on residents' willingness to purchase low-carbon vegetables using a conditional value assessment approach. The significant effects of gender, education level, low carbon awareness, and habits of purchasing vegetables in traditional markets, large supermarket chains, and community supermarkets on respondents' willingness to purchase low-carbon vegetables were investigated [43]. Through the construction of models and the use of different methods to study the intention to purchase goods and the attitudes and triggers that trigger consumers' willingness to pay a premium, several existing studies point to the influence of factors such as age, gender, marital status, occupational status, geographic location, and especially income and education [44] on different preferences. Estimating the level of consumer support and willingness to pay for low-carbon agricultural products [45, 46], while the household's willingness to accept equals the maximum individual willingness to accept in the case of income sharing [47, 48].

The purchase decision process is a decision-making process in which consumers analyze and evaluate a product internally and then make a choice to buy it [49–51]. The process is systematic and involves the generation of needs and motivations, the selection of purchase options, the implementation of the purchase behavior, and the postpurchase evaluation. There are five stages to a purchase decision, namely, the awareness of need stage, the information gathering stage, the evaluation decision stage, the behavior generation stage, and the product evaluation stage, and each of these stages is influenced by a combination of factors. Buying behavior is usually determined by personal factors [52], product factors, market factors, and environmental factors. The behavioral decision-making process is divided into three main stages, namely, the rational consumption stage, the emotional consumption stage, and the emotional consumption stage. These stages tend to change with changes in the level of social productivity and the consumer's standard of living.

Many early scholars proposed some typical theories and models, such as the theory of rational behavior [53], theory of planned behavior [54], and technology acceptance model [55–57] to explain or predict consumers' online purchase intentions and behaviors, revealing the relationship between behavior, behavioral intentions, and their influences from social and psychological perspectives [58], but the more accepted theories and models nowadays are the value-based adoption model [59] and unified acceptance theory [55]. In contrast, purchase intention, as the likelihood that consumers are willing to purchase and consume a product, has been used by scholars studying marketing as a predictor of consumer buying behavior. Willingness to buy is a subjective tendency that determines and governs consumers' purchasing behavior decisions, and consumers make purchasing behavior decisions because the goods they buy can satisfy some of their needs. This is a psychological manifestation of consumption, and therefore, he considers purchase intention as a psychological tendency [60]. On this basis, some scholars have expanded the connotation of purchase intention to explain it. Purchase intention is composed of both rational and emotional reactions of consumers to goods [61]. It plays a positive role in guiding the production and operation activities of companies [62] in order to better influence consumers' purchasing behavior [63, 64]. And in fact, purchase intention is not the only determinant of consumer purchase behavior; there are many other factors that act together with purchase intention to guide consumers to generate consumer behavior [65]. The conditional value approach is one of the most widely used valuation methods in ecosystem service valuation and belongs to the non-market technology valuation method, which is applicable to the valuation of goods exchanged in the absence of real markets and alternative markets, and its core is to directly investigate and consult people's willingness to pay (WTP) for ecological services and express the economic value of environmental goods in terms of willingness to pay and net willingness to pay (NWTP).

## 3. Methodology and Research Design

### 3.1. Data Source and Measurement Scale

The research data in this paper were collected through a structured questionnaire, which was designed according to the content of the study into five sections: demographic characteristics, awareness of ecological agricultural products and purchase channels, factors influencing the purchase of ecological agricultural products, and consumer purchase experience and willingness to pay. The questionnaire was measured using the Likert 5-point scale method [10], with a score of 1-5 indicating the degree of satisfaction, with higher scores representing higher levels of agreement. A total of 601 respondents' personal data parameters such as gender, age, education level, occupation, and monthly household income were recorded and distributed to consumers for survey through an online questionnaire.

### 3.2. Sample and Data Collection

Basic research data were collected by distributing questionnaires to Harbin City, Heilongjiang Province, the capital city of northern China, and a total of 601 valid questionnaire data were received. The demographic characteristics of consumers were first analyzed, as detailed in Table 1.

The demographic characteristics of the consumers include information on gender, education level, marital status, age, and total monthly household income. The results show that about 43.93% of the respondents are male and the remaining 56.07% are female. There are differences in the education level of consumers in this survey, including 37 people with junior high school (and below) education, accounting for 0.62%; 76 people with high school education, accounting for 12.65%; 124 people with technical secondary, accounting for 20.63%; and 269 people with bachelor's degree, accounting for 44.76%. The number of people with master's degree or above was 95, accounting for 15.81%. Married consumers are the main group of agricultural products purchasing, which is representative for the study of consumers' willingness to purchase. The 366 consumers in this study have married marital status, accounting for 60.9%, and 39.1% are unmarried. The age distribution of the respondents varies greatly, with the most represented age group being between 21 and 30 years old, accounting for 40.77% of the sample respondents, followed by 51 to 60 years old, accounting for 17.64%, which are usually middle-aged and elderly people who are responsible for household chores and have a greater demand for agricultural products. The sample conducted a statistical survey of the respondents' intrahousehold situation, and the results showed that the largest number of households with 2-3 members (55.9%), the largest number of households without children (54.7%), and the number of elderly people with 2 members (33.44%). In addition, the sample also counted the occupational distribution and income of the respondents. The largest number of respondents (26.62%) worked in institutions (education, medical, scientific research, etc.), and most of them had a household income between 473 and 1100$, accounting for 38.94% of the total number of respondents in the sample.

Through the survey, it could be found that 339 respondents are the main members of the family shopping for food, accounting for 56.41%, while 408 people (67.89%) have actually purchased ecological agricultural products, accounting for a large proportion, which proves that the analysis of the willingness of the interviewed group to purchase agricultural products is representative and scientific; 71.71% of consumers prefer to use farmers' markets, supermarkets 71.71% of the consumers prefer farmers' markets, supermarkets, and traditional e-commerce websites as traditional purchasing locations. There are differences in the results of the survey on the satisfaction of daily purchased agricultural products, with the majority of consumers being more satisfied with the general agricultural products and average. According to the survey on ecological agricultural products, the number of people who have a certain degree of knowledge about ecological agricultural products is 448, accounting for 74.3%, while the remaining 25.7% of consumers have less knowledge, and there is still great room for improvement in the knowledge of ecological agricultural products; the statistical results on the channels of understanding ecological agricultural products show that the proportion of those who are recommended by common media (books, newspapers, etc.) and friends (recommended by social media, etc.) is the highest, accounting for 49.7%. This is greatly related to the rapid development of the Internet and the national publicity of ecological agricultural products.

### 3.3. Data Analysis

In order to test the reliability of the empirical data, a consistency analysis was performed using the statistical knowledge Cronbach's alpha coefficient. The alpha coefficient mainly tests the stability of the scale, and the level of reliability coefficient reflects the level of stability of the scale, and its reliability depends on each factor in the study. The value obtained was 0.916, which is higher than the critical value of 0.70, ensuring the reliability of the scale. Various statistical methods and techniques such as factor analysis, principal component analysis, regression analysis, and survival analysis were used to analyze the quantitative data collected by the structured questionnaire.

Prior to principal component analysis, the statistical results of the questionnaire on consumer attitudes toward ecological agricultural products were tested for data applicability using the Kaiser-Mayer-Olin (KMO) and Bartlett's test of sphericity [66]. The statistical coefficient of the KMO test was 0.943, which exceeded the established value of 0.6 recommended. Bartlett's test for sphericity was significant, indicating that the correlation between items was sufficiently high to be used for principal component analysis. The presence of covariance between the independent variables was measured using the variance inflation factor test (VIF method) and the tolerance method, and the serial correlation test was used to ensure the validity of the regression analysis.

By correlating the contribution of the factors, a gravel plot was drawn for their eigenvalues, and the number of main factor sequences was classified by observing the magnitude of the slope between the factors. The results shown in Figure 1 show that the slope from the second factor to the third factor begins to decrease and tends to level off. The third factor can be judged as the bending point. Based on the correlation principle that the factors on the gentle slope have small variance, the factor located on the second factor (with a larger slope) and its slope and with an eigenvalue greater than 1 was selected as the principal factor. Thus, the first two factors were used as the main factors for the SPSS regression analysis and were used as categorical data for the next analysis.

Next, principal component analysis was used as the extraction method, and the converged component matrix was finally obtained by normalized orthogonal rotation before the iteration and then factor rotation afterwards, as shown in Table 2.

The classification can be displayed according to the results in the table, and these indicators can be divided into two categories according to the high load. C1-C7 has a larger load on the first factor, and combined with the problem setting, ecological agricultural products are more nutritious, healthier, better in taste, higher in satisfaction, and safer than general agricultural products. It can be concluded that consumers support ecological agricultural products, so they are named as “willing to pay” consumers. C8-C15 has a large load on the second factor, and it is concluded that consumers are opposed to ecological agricultural products, so they are named as “unwilling to pay” consumers, which can reflect the existence of such consumers that may exist in ecological agricultural products. The lack of understanding of the phenomenon leads to the formation of opposition to consumption, these consumers are potentially huge consumption power in the market.

There are many factors that affect whether consumers choose to buy ecological agricultural products. In this paper, variables such as consumer basic information and socioeconomic attributes are selected as explanatory variables, and a binary logit-based consumer choice behavior model is established. Whether to choose ecological agricultural products is the dependent variable. Other variables are independent variables. In the model, the values of independent variables and dependent variables are multi-level.

For the independent variable *Y*, it is defined that those with willingness to pay are assigned a value of 1 (that is, to buy ecological agricultural products), and those without willingness to pay are assigned a value of 0 (that is, they are unwilling to buy ecological agricultural products). The dependent variable *X* = (*x*_1,_*x*_2⋯,_*x*_*n*,_) is an *n*-dimensional variable related to the occurrence of *Y*.When *x*_1,_*x*_2,_ ⋯ *x*_*n*_ takes a specific value, the probability of occurrence of *Y*( = 1) is

(1) $$\begin{array}{c} P_{r}=\left(Y=1\right)=\frac{\exp\left(B+\sum_{i=1}^{n}\beta_{i}X_{i}\right)}{1+\exp\left(B+\sum_{i=1}^{n}\beta_{i}X_{i}\right)}. \end{array}$$

Taking *Y* = 1, that is, willingness to pay, as the reference point, the regression results obtained by the application software SPSS 26.0 are shown in Table 3. Due to the large number of explanatory variables, the factors that do not have a significant impact are eliminated, and the factors with a significant impact are shown in Table 3.

The binary logit regression results show that for basic information of consumers, from the regression results, it can be seen that the marital status is married, the family size is large, and the number of children is significantly and positively correlated with whether they are willing to accept ecological agricultural products. Married people are more willing to accept ecological agricultural products. The survey shows that married people with a stable family life are happier. These people think more long-term, and they are more inclined to invest more in food quality and health care for the elderly and children. The educational level and age are significantly negatively correlated with whether they are willing to accept ecological agricultural products. To buy ecological agricultural products and their partners or parents are the main buyers, the cognition level of the highly educated respondents on ecological agricultural products is inconsistent with the actual consumption behavior. Therefore, their higher ecological cognition level and willingness to consume does not translate into actual purchase behavior. This conclusion is also consistent with the research results of Ping et al. [67] and Ming and Chang [68]. The older consumers have lower acceptance of ecological agricultural products, which may be mainly related to the popularity of ecological agricultural products in the middle-aged and young people.

For consumers' cognitive level and purchase experience, the regression results showed that purchase experience, understanding level, farmers' market purchase, Meituan (community group purchase), and monthly amount spent on agricultural products were significantly and positively correlated with whether they were willing to accept ecological agricultural products. Consumers who have purchased ecological agricultural products put forward higher requirements on the taste, quality, and safety of the agricultural products they purchase in the future. Consumers who have more exposure to ecological agricultural products, especially those who have had experience in purchasing ecological agricultural products, are more willing to choose ecological agricultural products again, and their demand for ecological agricultural products will increase. The higher consumers' knowledge of ecological agricultural products indicates that consumers with higher knowledge of the nutritional value of ecological agricultural products are more willing to buy ecological agricultural products. Consumers who buy ecological agricultural products in two types of channels, namely farmers' markets and Meituan (community group buying), are more willing to accept ecological agricultural products. The possible reason is that consumers think ecological agricultural products sold in farmers' markets are more reliable in terms of safety and quality, and they can see the freshness of ecological agricultural products at the time of purchase and avoid decay and occurrence of damage due to remote transportation from online shopping. However, consumers who choose Meituan (community group buying) may belong to people who are busy with their daily work and do not have free time to go to farmers' markets and other field purchases, so this way of shopping provides convenience for consumers. The more money they spend on agricultural products each month, the more they can accept ecological agricultural products, which means that ordinary agricultural products cannot meet consumers' demand for quality, so they are willing to choose safer and healthier ecological agricultural products to eat.

Through the survey on the factors that consumers think the price of ecological agricultural products is high (refer to Figure 2 and Table 4), more than 85% of the consumers consider that the price of ecological agricultural products is high for the reason that the packaging increases the cost; the yield is low; the production cost, the labor cost, and the circulation cost increase; and the ecological agricultural products are of better quality; among these factors, the better quality of ecological agricultural products has the greatest influence on the high price of ecological agricultural products. These factors are very important for consumers to purchase ecological agricultural products, and they are the key factors that affect whether consumers buy them again or not. Based on this, in order to further investigate the consumers' payment premium for ecological agricultural products, the logit model in survival analysis is applied to estimate the consumers' payment premium for ecological agricultural products, and the survival function of WTP can be derived based on the parameter values, and further the expected value of WTP can be obtained.

### 3.4. Model Construction

The product chosen for this study is ecological rice because rice is the most important food in the diet of people in China and the world, and ecological rice is highly representative as an important part of ecological agricultural products in China. Applying the logit model in survival analysis to estimate the consumer's payment premium for ecological agricultural products, the survival function of WTP can be derived from the parameter values, and further, the expected value of WTP can be obtained. The probability function when the response case of consumer's response to the initial bid amount *T* is positive is determined as the survival function. The survival function *S* and the distribution function *G* are related by *S* = 1 − *G*. If the distribution function *S* is assumed to be normally distributed, the survival function can be expressed as

(2) $$\begin{array}{c} S\left(T\right)=1-\emptyset \left[\frac{T-\delta }{\gamma }\right], \end{array}$$

where *δ* is the scale parameter and *γ* is the shape parameter.

At this point, the resulting likelihood function is

(3) $$\begin{array}{c} \ln L=\underset{i=\text{YES}}{\sum }\ln S\left(T\right)+\underset{i=\text{NO}}{\sum }\ln\left(1-S\left(T\right)\right), \end{array}$$

where YES represents the number of consumers who responded affirmatively to the prompted amount and NO represents the number of consumers who responded negatively to the prompted amount.

(4) $$\begin{array}{c} \log h\left(T\right)=\alpha \log T+\beta_{0}+\beta_{1}X_{1}+\cdots +\beta_{i}X_{i}. \end{array}$$

In the above equation, *α* = 1/(*γ* − 1), *β*_0_ is a constant term, and *β*_1_, *β*_2_, ⋯*β*_*i*_(*i* = 1, 2, ⋯*n*) is the coefficient of influence factor *X*_1_, *X*_2_, ⋯*X*_*i*_(*i* = 1, 2, ⋯*n*).

In order to derive the final magnitude of consumers' willingness to pay, the logit model in survival analysis is applied to estimate consumers' payment premium for ecological agricultural products, and the survival function of WTP can be derived based on the parameter values to further obtain the expected value of WTP.

The survival function of the logit model fitted to the survival data is

(5) $$\begin{array}{c} S\left(\text{WTP}\right)=1-F\left\{\frac{\left(\log\text{WTP}-\delta \right)}{\gamma }\right\}. \end{array}$$

The WTP expectation is calculated by the formula:

(6) $$\begin{array}{c} E\left(\text{WTP}\right)=\int_{0}^{\text{WTP}}\left\{1-\frac{\log\left(\log\text{WTP}-\delta \right)}{\gamma }\right\}d\text{WTP}. \end{array}$$

After reviewing the existing studies on double-bounded dichotomies and thinking deeply about them [69, 70], the above five versions of the questionnaire were designed (as shown in Table 5), and the initial bid values of the double-bounded dichotomous questionnaire were set at five values: 5, 20, 35, 50, and 65. Since the expected value of the respondents' WTP is related to their own income level, the willingness to pay needs to be bounded, and a right intercept of the WTP and its distribution at the initial maximum bid value is the most reliable method. In this paper, the WTP_max_ is 65%, and it is brought into the average willingness to pay calculation formula, and the survival analysis function is run through the program, and the scale parameters and shape parameters of the logit model are calculated by using SAS software to obtain *δ* = 0.139 and *γ* = 0.361, and the expected value of WTP is 24.9466 when brought into the model, which means that consumers are willing to pay more for ecological agricultural products than general agricultural products 24.95%. Using the writing program to obtain the impact results of each attribute, the model results of survival analysis were obtained by running the logit model through SAS. The impact of each attribute variable on willingness to pay can be obtained based on the analysis in the table, as shown in Table 6 below.

Regarding basic information, gender, education level, marital status, age, monthly household income, number of children in the household, and number of elderly in the household had a significant effect on willingness to pay. Gender has a significant effect on willingness to pay and is positively correlated, indicating that women are more willing to pay a premium for ecological agricultural products, and women tend to be more willing to choose ecological agricultural products as the main role of household chores in the family. Marital status is positively correlated with willingness to pay, indicating that married consumers are more willing to pay extra price for ecological agricultural products; the number of children in the household is significantly and positively correlated with willingness to pay, and families with more children are more willing to pay more price for ecological agricultural products. The number of elderly people in the household is positively correlated with willingness to pay, and the more elderly people in the household, the more likely the household is to pay a premium price for ecological agricultural products. Educational attainment, age, and monthly household income were negatively correlated with willingness to pay for ecological agricultural products, indicating that consumers with higher educational attainment were less willing to pay a premium for ecological agricultural products, and older consumers were less willing to pay an extra price for ecological agricultural products. Consumers with higher monthly household income were not willing to pay a premium for ecological agricultural products. More than 85% of consumers believed that the high price of ecological agricultural products was due to the increased cost of packaging, low yield, increased production, labor and distribution costs, and better quality of ecological agricultural products. Among these factors, better quality of ecological agricultural products had the greatest impact on the high price of ecological agricultural products.

Regarding the factors influencing the purchase of ecological agricultural products, the two main factors FAC1-1 (supportive) and FAC2-1 (opposed) extracted by factor analysis had a more significant effect on willingness to pay. Among them, FAC1-1 is positively correlated with willingness to pay, indicating that consumers with positive attitudes toward ecological agricultural products are more willing to pay extra price for ecological agricultural products, and the results are also consistent with the actual; FAC2-1 is negatively correlated with willingness to pay, indicating that consumers with negative attitudes toward ecological agricultural products are not willing to pay premium price for ecological agricultural products, and this part of consumers are potential future buyers of consumers of ecological agricultural products.

## 4. Analysis of Results

Based on the data analysis and model results, it could be concluded that consumers' marital status, number of children in the household, ecological agricultural products purchasing experience, knowledge of ecological agricultural products, channels of purchasing ecological agricultural products, education level, age, and household size have significant influence on choosing ecological agricultural products.

1. Marital status has a significant positive correlation with the purchase of ecological agricultural products. Married consumers, as the main purchasers of ecological agricultural products, have a greater tendency to purchase ecological agricultural products, so they are more willing to purchase ecological agricultural products, while children, as the main concern group of families and even society, parents pay much attention to them in terms of food safety and food health. The results show that there is a significant positive correlation between the number of children and the purchase of ecological agricultural products, which is consistent with the actual situation
2. Consumers who have purchased ecological agricultural products are positively related to their purchase intentions, which is also consistent with consumers' choice behavior. Consumers who have not purchased ecological agricultural products have certain limitations in their knowledge and they cannot have a comprehensive understanding of them
3. Consumers with higher understanding of ecological agricultural products are more willing to accept ecological agricultural products because they are aware of the nutritional value of ecological agricultural products and the ecological value in the social sense, thus prompting their purchase
4. In terms of the channel of understanding ecological agricultural products on choosing ecological agricultural products, consumers who buy ecological agricultural products at farmers' markets and Meituan and community group purchases are more willing to accept ecological agricultural products, while the opposite result exists for consumers who buy agricultural products at other locations and tend to be reluctant to accept ecological agricultural products
5. The higher the monthly consumption of agricultural products, the greater the tendency of households to choose ecological agricultural products. The likely situation is that consumers have average feelings about the general agricultural products they buy, which cannot meet their daily needs for agricultural products, and therefore choose to buy higher quality ecological agricultural products. This is consistent with their findings [71]

Education level, age, and household size were significantly and negatively correlated with consumers' purchase of ecological agricultural products. Although consumers with higher education level have more rational judgment and clearer understanding of ecological agricultural products and thus are more inclined to choose ecological agricultural products, the results show a negative correlation, which may be due to the fact that those with higher education level have less time and energy to shop for ecological agricultural products due to their more important work in society, while their partners or parents act as the main purchasers. The level of awareness of ecological agricultural products and the actual consumption behavior of the respondents with high education are nonconsistent; therefore, their higher level of ecological awareness and consumption intention do not translate into actual purchasing behavior. This finding is also consistent with the findings of Ping [67] and Ming and Chang [68]. The lower acceptance of ecological agricultural products by the older consumers may be mainly associated with the fact that the popularity of ecological agricultural products is mostly among the middle-aged and young people. The results of the study showed that family size was significantly and negatively associated with willingness to pay for ecological agricultural products, which may be due to the fact that most of the consumers with large family size are married and prefer to choose common agricultural products considering the economic aspects because the price of ecological agricultural products is higher than that of common agricultural products.

The two main factors FAC1-1 (supportive) and FAC2-1 (opposed) extracted by factor analysis had a relatively significant effect on willingness to pay. Among them, FAC1-1 is positively correlated with willingness to pay, indicating that consumers with positive attitudes toward ecological agricultural products are more willing to pay extra price for ecological agricultural products, and the results are also consistent with the reality; FAC2-1 is negatively correlated with willingness to pay, indicating that consumers with negative attitudes toward ecological agricultural products are not willing to pay extra price for ecological agricultural products, and if this group of consumers can in the future If this group of consumers can realize the significance of ecological agricultural products for health and social sustainability in the future, they are likely to switch to buying ecological agricultural products.

Among all the questions on the reasons for refusing to buy ecological agricultural products, the most common reasons are that consumers believe that general agricultural products are sufficient to meet their current daily needs and that ecological agricultural products are too expensive, accounting for 26.89% and 28.05%, respectively. Some consumers think that the market supervision department should strengthen the supervision of ecological agricultural products.

## 5. Conclusion and Outlook

This paper takes ecological agricultural products as the research object, collects information about 601 consumers' cognitive status and willingness to pay for ecological agricultural products in Harbin through an online questionnaire survey, analyzes the factors influencing their purchase of ecological agricultural products by establishing a binary logit consumer choice behavior model, and analyzes the factors influencing consumers' payment premium for ecological agricultural products through survival and finally calculates the average payment premium of consumers premium; the following conclusions are mainly obtained.

Consumers' knowledge of ecological agricultural products is not high, and there is still more room for consumers' awareness of ecological agricultural products and sellers' publicity and popularization. By broadening consumers' access to information, a portion of consumers who are dissatisfied with the existing general agricultural products may be converted into consumption power to purchase ecological agricultural products; more than half of the consumers who have never purchased agricultural products are the key potential consumers of ecological agricultural products. Regarding the knowledge of ecological agricultural products, 71.8% of consumers do not know much about ecological agricultural products and still have cognitive bias, thinking that ecological agricultural products are only general agricultural products beautifully packaged and sold at high prices. However, through the purchase channels, we can find that with the popularity of Internet and the important role played by cell phones in daily life, it has become a mainstream channel to learn about ecological agricultural products through Internet.

Based on the regression results of the survival analysis model, the factors that influence consumers' willingness to pay were analyzed. For basic information: consumers who often go to supermarkets are willing to pay more for ecological agricultural products; consumers who are less satisfied with the general agricultural products they buy are willing to pay more for ecological agricultural products; consumers who have bought ecological agricultural products and know more about ecological agricultural products are also willing to pay more for ecological agricultural products; consumers who learn about ecological agricultural products through friends and the Internet are also willing to pay more for ecological agricultural products. Consumers who learn about ecological agricultural products through friends and the Internet are also willing to pay extra for ecological agricultural products. Consumers who are optimistic and supportive of ecoproducts are more willing to pay, while those who are opposed to eco-products are less willing to pay, and the results are consistent with reality. Not the main member of the family is more inclined to accept ecological agricultural products; women and single are relatively more willing to accept ecological agricultural products. Age, however, is negatively correlated with the degree of acceptance. Meanwhile, consumers with higher education level and higher income are relatively more willing to pay. Finally, consumers' payment premium for ecological agricultural products is 24.95%, which means that consumers in Harbin can accept that purchasing ecological agricultural products is 24.95% more expensive than general agricultural products, then the market price of ecological agricultural products is suggested to be about 24.95% more expensive than general agricultural products.

At this stage, consumers' understanding of ecological agricultural products is limited and still at the level of superficial awareness and less exposure. Consumers' perception of cost performance directly determines consumers' attitude and selection behavior, and the higher the level of perception, the easier consumers are to make acceptance behavior. Consumers' awareness of ecological agricultural products largely depends on the publicity power of the society. With the popularity of the Internet and the important role of cell phones in daily life, the market can increase the degree of purchase by improving online information propaganda and refreshing the traditional impression of ecological agricultural products. In addition, with the development of online selling of ecological agricultural products in full swing, choosing e-commerce form for online selling is another new way.

The role of market promotion remains the focus of the future. The direction of government support often represents the future direction of industrial development, and the credibility and policy support of the government can effectively promote the development of special ecological agricultural products. Ecological agricultural products manufacturers and farmers need to better cater to the diverse needs of consumer groups, so as to lock in target consumers and finally achieve accurate marketing. To do so, consumers can directly access information about enterprises and ecological agricultural products, which provides convenience for enterprises to enhance their visibility and promote ecological agricultural products brands, and it is more conducive to the realization of international brand marketing of agricultural products.

In this paper, a comprehensive statistical approach is used to study the influencing factors of consumers' purchase of ecological agricultural products, and an in-depth analysis of the reasons for consumers' refusal to pay is conducted to arrive at the most realistic willingness to pay and the related influencing factors, and a survival analysis model is constructed to study the level of premium payment. In this study, only the selected factors were investigated and studied to derive the influence of these factors on consumers' purchase of ecological agricultural products. The next study will continue to focus on other aspects of factors that may have an impact on consumers' purchase of ecological agricultural products, such as marketing methods and government regulation, to further explore the extent of the role of other influencing factors, so as to achieve on-demand supply. In addition, the location of this study is Harbin City, Heilongjiang Province, which is representative but may have some geographical limitations. Therefore, in order to achieve the universality and extensiveness of the research results, more regions will be studied in the future, so as to provide a basis for the marketing of ecological agricultural products producers and government policies.

## Figures and Tables

**Figure 1:** Gravel figure.

**Figure 2:** Consumers' recognition of the premium of ecological agricultural products.

**Table 1:** Statistical table of basic information of respondents.

Basic information	Content	Number of respondents	Proportion
Gender	Male	264	43.93%
	Female	337	56.07%

Education	Junior high school and below	37	0.62%
	High school	76	12.65%
	Technical secondary	124	20.63%
	Bachelor	269	44.76%
	Master/PhD	95	15.81%

Marital status	Married	366	60.9%
	Unmarried	235	39.1%

Age (years)	≤20	23	0.38%
	21-30	245	40.77%
	31-40	94	15.64%
	41-50	97	16.14%
	51-60	106	17.64%
	≥60	36	0.6%

Occupation	Retirees	71	11.81%
	Party and government	66	10.98%
	Public institution organs	160	26.62%
	State-owned enterprises	96	15.97%
	Foreign/joint venture/private enterprise	66	10.98%
	Self-employed/others	142	23.63%

Household income/month ($)	≤472	76	12.65%
	473-786	125	20.8%
	787-1,100	109	18.14%
	1,101-1,415	104	17.3%
	1,416-1,730	75	12.48%
	≥1,731	112	18.64%

Household size	1	42	0.7%
	2-3	336	55.91%
	4-5	165	27.5%
	6-7	55	0.92%
	≥8	3	0.05%

Number of children in the family	0	329	54.74%
	1	191	31.78%
	2	63	10.5%
	3	11	0.18%
	≥4	7	0.17%

Number of elderly in the household	0	175	29.12%
	1	165	27.45%
	2	201	33.44%
	3	33	0.55%
	≥4	27	0.45%

**Table 2:** Component matrix after rotation.

Factors	Ingredient 1	Ingredient 2	Code
Satisfaction with purchased ecological agricultural products is better than general agricultural products	0.613	0.254	C1
Ecological agricultural products are more nutritious	0.757	0.182	C2
Ecological produce tastes better	0.628	0.382	C3
Eating ecological agricultural products is healthier	0.769	0.213	C4
We buy ecological agricultural product specifically for children because it is healthier	0.702	0.312	C5
We buy ecological agricultural product specifically for the elderly because it is healthier	0.663	0.390	C6
Ecological agricultural products are safer than ordinary agricultural products	0.664	0.386	C7
Ecological agricultural products do not play a role in environmental protection	0.448	0.531	C8
Ecological agricultural products are no fresher than ordinary agricultural products	0.406	0.578	C9
The types of ecological agricultural products are not as complete as general agricultural products	0.360	0.650	C10
Choose to buy ecological agricultural products online because it is inconvenient to go to the supermarket or farmers market	0.125	0.688	C11
The quality of ecological agricultural products cannot be guaranteed	0.288	0.671	C12
The frequency of daily purchase of ecological agricultural products is not as high as that of general agricultural products	0.309	0.666	C13
The packaging of ecological agricultural products is not very practical	0.226	0.705	C14
The price of ecological agricultural products in the market is too high	0.382	0.467	C15

**Table 3:** Binary logit regression parameter results.

Variable	B	Std. error	Wald	*P*	Exp(*B*)	95% confidence limit	
						Lower limit	Upper limit
(Constant)	-0.572	1.039	0.303	0.582	0.564		
Education level	-0.241	0.122	3.895	0.048	0.786	0.619	0.998
Marital status	1.932	0.365	28.055	0.001	6.902	3.377	14.107
Age	-0.706	0.109	42.108	0.001	0.494	0.399	0.611
Household size	-0.471	0.168	7.898	0.005	0.624	0.450	0.867
Number of children in the family	0.549	0.163	11.323	0.001	1.731	1.257	2.383
Purchase experience	1.246	0.258	23.346	0.001	3.477	2.097	5.763
Level of understanding	0.257	0.111	5.420	0.020	0.773	0.623	0.960
Farmers' market	1.442	0.242	35.631	0.001	4.230	2.634	6.792
Meituan, community group buying	0.816	0.285	8.209	0.004	2.262	1.294	3.955
Spent on purchasing agricultural products/month	0.202	0.09	5.058	0.025	1.224	1.026	1.461

**Table 4:** Findings on the causes of high prices of ecological agricultural products.

Premium question settings	Number of accredited	Number of unaccredited	Code
Packaging increases costs	513	88	D1
Low yield	537	64	D2
Increase in production costs	545	56	D3
Increase in labor costs	527	74	D4
Increase in circulation costs	524	77	D5
Better quality	556	45	D6

**Table 5:** Basic statistics of ecological agricultural products CVM questionnaire.

Type of questionnaire	Initial bid value	Lower bid value	Upper bid value	Frequency
A	5	0	10	117 (19.47%)
B	20	10	35	119 (19.80%)
C	35	20	50	118 (19.63%)
D	50	35	65	120 (19.97%)
E	65	50	80	127 (21.13%)
Total: 601 (100%)				

**Table 6:** Survival analysis regression results.

Parameters	Estimate	Std. error	95% confidence limit		Chi-square	*Pr* > chi‐square
Intercept	27.2631	3.2815	20.8314	33.6948	69.02	<0.0001
Gender	2.4510	0.6626	1.1524	3.7497	13.68	0.0002
Education level	-1.1838	0.3195	-1.8100	-0.5576	13.73	0.0002
Marital status	11.7820	0.8727	10.0716	13.4924	182.28	<0.0001
Age	-4.5217	0.1951	-4.9040	-4.1393	537.23	<0.0001
Occupation	-0.0410	0.2554	-0.5417	0.4596	0.03	0.8724
Monthly household income	-0.6788	0.2136	-1.0975	-0.2601	10.10	0.0015
Household size	-0.1454	0.5293	-1.1827	0.8919	0.08	0.7835
Number of children in the family	2.8097	0.3010	2.2197	3.3996	87.14	<0.0001
Number of elderly people in the family	1.4553	0.3393	0.7903	2.1203	18.40	<0.0001
FAC1 supportive	2256.332	324.1503	1621.009	2891.655	48.45	<0.0001
FAC2 opposed	-56.5950	5.8252	-68.0123	-45.1778	94.39	<0.0001
Scale	1	0.0000	1	1		

## Data Availability

Data for this study are securely kept by the principal investigator and will be made available upon request.
